# Expression and Clinicopathological Significance of SOX11 in Small-Cell Lung Cancer

**DOI:** 10.1155/2022/1707914

**Published:** 2022-03-30

**Authors:** Wang Xinli, Wang Lixiao, Ding Baoqi, Huang Hu, Zhang Qiang

**Affiliations:** ^1^Department of Pathology, The Second Affiliated Hospital of Shandong First Medical University, Taian City, Shandong Province, China; ^2^Shandong First Medical University, Taian City, Shandong Province, China

## Abstract

**Objective:**

This study aims to investigate the expression of neuronal transcription factor SOX11 in small-cell lung cancer (SCLC) and compare it with the expression of CD56 (nerve cell adhesion molecule), synaptophysin (Syn), chromogranin A (CgA), and thyroid transcription factor-1 (TTF-1) to explore the application value of SOX11 in the pathological diagnosis of SCLC.

**Methods:**

Immunohistochemical methods were used to detect the expression of SOX11, TTF-1, CD56, Syn, and CgA in 120 lung tumor tissues, and experimental results were analyzed using SPSS23.0 statistical software.

**Results:**

Immunohistochemical results showed that in the 120 lung tumor samples, SOX11 was highly expressed in SCLC and localized to the nucleus, with low or no expression in control carcinoid/lung neuroendocrine tumors, lung adenocarcinomas, and lung squamous cell carcinomas. Statistical analysis results revealed the following points. First, the expression of SOX11 was closely related to the tumor histological type. The expression of SOX11 in SCLC (positive rate of 63.33%) was significantly higher than that in carcinoid/neuroendocrine tumors (positive rate of 12.50%), lung adenocarcinoma (positive rate of 0%), and lung squamous cell carcinoma (positive rate of 0%). Second, immunohistochemical investigation of 60 SCLC cases revealed that the highest positive rates of CD56, TTF-1, and Syn, respectively, were 93.33 percent, 95 percent, and 86.67 percent. SOX11 also exhibited high sensitivity (0.633) and specificity (0.875) in SCLC. The positive rates of SOX11 and CgA were 63.33% and 50.00%, respectively. Statistical results revealed that the positive rate of CgA had no significant difference (*P* > 0.05). Lastly, the combined use of antibodies SOX11, CgA, CD56, Syn, and TTF-1 was more beneficial to improving the diagnosis rate of SCLC than the single use of one or two antibodies.

**Conclusion:**

The expression of SOX11 in different histological types of lung tumors differs considerably. SOX11 is highly expressed in SCLC. SOX11 can be used as a beneficial supplement to the combination of classical neuroendocrine markers and in combination with CgA, CD56, Syn, and TTF-1 to assist in the diagnosis of SCLC.

## 1. Introduction

The incidence and mortality of lung cancer have increased rapidly in China in recent years. As a high-grade neuroendocrine tumor, small-cell lung cancer (SCLC) has a worse prognosis than non-small-cell lung cancer (NSCLC) because of its acute progression and early metastasis of lymph nodes and distant organs, and the mortality rate can reach 90% [1]. NSCLC usually requires surgery, whereas SCLC is sensitive to chemotherapy and radiotherapy [2]. Therefore, in the histological classification of lung cancer, distinguishing other types of lung cancer from SCLC is crucial and the key to selecting the appropriate treatment method for patients with lung cancer. This work relies on the precise diagnosis of pathologists. In practice, patients with SCLC exhibit early clinical symptoms. Through early accurate diagnosis, clinical staging, and comprehensive evaluation, the best treatment plan is selected for active treatment as soon as possible, and patients can survive for a long time [3].

However, the diagnosis of SCLC remains difficult in current clinical and pathological work. Tissue structure and cell morphology are often difficult to identify due to insufficient tissue fixation, improper specimen handling, heavy tissue extrusion, poor tissue adhesion, and tissue necrosis, making SCLC difficult to distinguish from other diseases, such as non-small-cell carcinoma, carcinoid, large-cell neuroendocrine carcinoma, basal-like squamous cell carcinoma, non-Hodgkin's lymphoma, metastatic breast cancer, and chronic inflammation. Therefore, immunohistochemistry is crucial in the pathological diagnosis of SCLC.

The SOX protein family is a key transcription factor for many developmental processes [4] and common diseases [3]. The important roles of SOX factors in the proliferation, migration, invasion, and metastasis of various tumor cells have been widely studied in recent years. As an important transcription factor that regulates neurogenesis, SOX11 can be used as a new neuroendocrine index to assist in the diagnosis of SCLC, but only a few studies have been conducted at home and abroad.

On this basis, this study randomly selected 120 patients with lung puncture and radical surgery in our hospital from 2019 to 2021 as the research subjects. The aim was to investigate the expression of SOX11 in SCLC and analyze its clinicopathological value.

## 2. Materials and Methods

### 2.1. General Information

A total of 120 paraffin specimens of lung tumors (including 60 cases of SCLC) were used. The HE sections of the cases were read by two senior attending physicians attending. The corresponding wax blocks were selected from the wax block library of the Department of Pathology and sliced continuously. SOX-11 antibody immunohistochemical staining was performed on the pathological sections of the 120 cases, and CD56 (nerve cell adhesion molecule), thyroid transcription factor-1 (TTF-1), synaptophysin (Syn), and chromogranin A (CgA) antibody immunohistochemical staining were performed on the pathological sections of the 60 cases of SCLC. Our study obtained patient or family consent and was approved by the hospital ethics committee.

### 2.2. Main Experimental Reagents

SOX11, TTF-1, CD56, Syn, and CgA were ready-to-use antibodies and purchased from Fuzhou Maixin Biotechnology Development Co., Ltd.

### 2.3. Experimental Instruments and Equipment

The experimental equipment were a paraffin microtome (RM2235, Leica Microsystems, Inc.), a microtome (YT-7FB, Leica Microsystems, Inc.), an automatic immunohistochemistry machine (Benchmark XT, Ventana Medical Systems, Inc.), and an optical microscope (ECLIPSE Ni-U, Nikon Corporation, Japan).

### 2.4. Immunohistochemical Staining

The thickness of the paraffin block section was 3 *μ*m. Each immunohistochemical section had the corresponding positive and negative control tissues attached to the far-right end of the slide. Each section was stained using a Benchmark XT automatic immunohistochemical machine. After dehydration, transparency, and mounting, the slides were placed under a microscope for observation.

### 2.5. Interpretation of Results

SOX11 and TTF-1 were positive in nuclear immunostaining, CD56 positive was located in the cytoplasm and cell membrane, and Syn and CgA were positive in cytoplasmic staining. If more than 1% of tumor cells are stained, then the immunohistochemical results can be considered positive [5]. The results were observed with the double-blind method and evaluated by two senior pathologists at the attending level and above to ensure the accuracy of the results.

### 2.6. Statistical Analysis

SPSS 23.0 (IBM Corporation, Armonk, NY) software was used, the count data were expressed in percentage (%), and a hypothesis test was performed through the *χ*^2^ test. When the two-tailed *P* value was less than 0.05, the difference was considered statistically significant.

## 3. Results

A total of 120 cases of lung tumors were selected; the total cases included 60 cases of small-cell carcinoma, 16 cases of carcinoid/neuroendocrine tumor, 20 cases of adenocarcinoma, 20 cases of squamous cell carcinoma, 2 cases of adenosquamous cell carcinoma, 1 case of carcinosarcoma, and 1 case of large-cell neuroendocrine carcinoma. Considering that the sample size of adenosquamous cell carcinoma, carcinosarcoma, and large-cell neuroendocrine carcinoma was very small but could not be excluded in the statistical analysis, we only analyzed and summarized the data of 116 patients in four cases: SCLC, carcinoid/neuroendocrine tumor, lung adenocarcinoma, and lung squamous cell carcinoma.

### 3.1. Relationship between the Expression of SOX11 and Tumor Histological Types

The positive rate of SOX11 in SCLC was higher than that in lung neuroendocrine tumor, lung adenocarcinoma, and lung squamous cell carcinoma. Among the 60 cases of SCLC, 38 were positive for SOX11 (63.33%). Among the 16 cases of carcinoid/neuroendocrine tumors, only 2 were positive for SOX11 (12.50%). SOX11 was negatively expressed in all cell carcinomas in the 20 cases of lung adenocarcinoma and 20 cases of lung squamous cell carcinoma (Table 1).

### 3.2. Comparison of Positive Rates of Antibodies SOX11, TTF-1, CD56, Syn, and CgA in SCLC

In the 60 cases of SCLC, the positive rates of antibodies CD56, TTF-1, and Syn were the highest at 93.33%, 95%, and 86.67%, respectively. The positive rates of SOX11 and CgA were 63.33% and 50.00%, respectively (Table 2 and Figure 1).

The chi-square test showed that although the positive rate of SOX11 was lower than that of CD56, TTF-1, and Syn, the positive rate of SOX11 was not significantly different from that of CgA (*Χ*^2^ = 0.862, *P* = 0.458). SOX11 also showed higher sensitivity (0.633) and specificity (0.875) in SCLC than the other neuroendocrine antibodies. This result indicates that SOX11 can display a certain degree of neuroendocrine differentiation and can be combined with CgA, CD56, TTF-1, Syn, and other markers for the pathological diagnosis of SCLC.

### 3.3. Expression Distribution of Antibodies SOX11, TTF-1, CD56, Syn, and CgA in SCLC

The specific expression distribution of the five antibodies in SCLC is summarized in Table 3.

In 31 of the 60 SCLC cases (51.60%), the three traditional neuroendocrine tumor markers, namely, CD56, Syn, and CgA, were not fully expressed (i.e., they were not simultaneously positive). Of the 31 SCLC cases, 17 (54.8%) were positive for the antibody SOX11. These statistical results indicate that the combined use of four or five antibodies is more beneficial to improving the diagnosis rate of SCLC than the single use of one or two antibodies.

## 4. Discussion

Pathological diagnosis is the gold standard for diagnosing SCLC. Given that the standard treatment for SCLC is radiotherapy and chemotherapy, obtaining large surgical specimens of SCLC is difficult. Generally, only a small amount of tissues can be obtained for pathological diagnosis through lung tissue puncture biopsy, lung brush examination, and lung lavage cytology [6]. The microscopic histological characteristics of SCLC are as follows: round-, oval-, or spindle-shaped cells; lack of cytoplasm; dense staining of nucleus; fine dispersion of nuclear chromatin; no obvious nucleolus; clearly visible nuclear division; and severe tissue extrusion. Thus, SCLC is easily confused with lymphoma, chronic inflammation, and other diseases. Moreover, the sample volume and tumor component are too small, so providing a definitive diagnosis is difficult. Therefore, in clinical pathological work, immunohistochemistry is essential for confirming the epithelial or neuroendocrine phenotype of tumor cells.

At present, the most commonly used immunohistochemical antibody combination for the clinicopathological diagnosis of SCLC is TTF-1 combined with neuroendocrine markers, including CD56, Syn, and CgA.

TTF-1 is expressed in SCLC in 85%–90% of cases [7]. Studies have shown that TTF-1 may become a biomarker for predicting the efficacy and prognosis of SCLC treatment [8]. However, Zheng et al. [9] found that SCLC and poorly differentiated lung adenocarcinoma have immune responses to TTF-1, but TTF-1 alone cannot distinguish the two.

As a neural cell adhesion molecule, CD56 is specifically expressed in neuroendocrine tissues and tumors. Studies have shown that CD56 is highly sensitive to SCLC, and even in heavily squeezed or decalcified biopsy specimens, CD56 can exhibit consistent, diffused, strong cytoplasmic staining [10]. However, CD56 is also expressed in NK cells, activated T cells, and lymphocytes [11]. These cells are morphologically similar to SCLC cells in HE sections and not easily distinguished.

Syn is expressed in neuroendocrine cells in normal human tissues [12]. Studies have shown that in carcinoid and classical SCLC cell types, Syn may be a more sensitive immunohistochemical marker for neuroendocrine differentiation than CgA [13].

CgA is the most specific marker of neuroendocrine differentiation [14]. It is ubiquitous in neuroendocrine tissues. Studies have found that SCLC only expresses CgA in a small number of cases [15]. Clinical work has also shown that the expression rate of CgA in SCLC is not ideal.

Although the classical antibodies CD56, Syn, and CgA are a good group of SCLC immunohistochemical combinations, their expressions are often not completely consistent in actual diagnosis. According to literature, about 10% of SCLCs are negative for CD56, Syn, and CgA [16].

Several studies have reported that neuroendocrine phenotype is a prognostic factor for SCLC, and it can provide an effective basis for the diagnosis and individualized treatment of SCLC [17]. Therefore, new neuroendocrine tumor markers need to be identified to assist in the diagnosis of SCLC.

As a member of the SOX family, SOX11 is a neurogenic transcription factor. Studies have revealed that it plays a key role in embryonic neurogenesis and neuronal cell fate [18]. Research on SOX11 has recently shifted its focus from the role of SOX11 in embryogenesis and development to its role in diseases. In particular, the role of SOX11 in carcinogenesis has become a major concern.

A previous study found a significant expression of SOX11 in SCLC (68%) [19]. SOX11 appears to be a valuable diagnostic and prognostic marker for aggressive neuroendocrine tumors [20]. Therefore, the use of SOX11 by immunohistochemistry can improve the diagnosis of SCLC and aggressive neuroendocrine lung cancer subgroups, which is beneficial for clinical risk stratification and selection of appropriate treatment methods.

Although several studies have shown that the expression of SOX11 is increased in lung neuroendocrine tumors, the expression and clinical importance of SOX11 in SCLC have rarely been explored. This study proves that SOX11 is highly expressed in SCLC, and it can be used as a beneficial supplement to the combination of neuroendocrine markers, thereby improving the diagnosis rate of SCLC. Early clinical diagnosis and treatment of SCLC are crucial for improving the survival rate of patients.

Although this study provides a rare analysis of the application of SOX11 in SCLC at home and abroad, it is based on a limited number of cases. Thus, additional data from other researchers are needed to support the results.

## Figures and Tables

**Figure 1:** (a) SCLC tumor cells are oval, short, and spindle-shaped. They have hyperchromatic nuclei but no obvious nucleoli, and the tumor cells grow in sheets with extrusion of HE ×200; (b) CD56-positive expression via diffused cytoplasmic membrane staining and IHC ×200; (c) TTF-1-positive expression, nuclear staining, and IHC ×200; (d) Syn-positive expression, cytoplasmic staining, and IHC ×200; (e) CgA-positive expression, cytoplasmic staining, and IHC ×200; (f) SOX11-positive expression, nuclear staining, and IHC ×200.

**Table 1:** Expression of SOX-11 in lung tumors of different histological types.

Tumor histological type	SOX11 expression		Positive rate	*P* value
	Positive	Negative		
SCLC	38	22	63.33%	
Carcinoid/neuroendocrine tumor	2	14	12.50%	0.001
Adenocarcinoma	0	20	0	<0.001
Squamous cell carcinoma	0	20	0	<0.001

**Table 2:** Comparison of positive rates of SOX11, TTF-1, CD56, Syn, and CgA in SCLC.

Antibody	Number of cases	Number of positive cases	Number of negative cases	Positive rate	*X* ^2^ value	*P* value
SOX11	60	34	26	56.67%		
CD56	60	56	4	93.33%	15.908	<0.001
TTF-1	60	55	5	91.67%	13.811	<0.001
Syn	60	52	8	86.67%	8.711	0.006
CgA	60	33	27	55.00%	0.862	0.458

**Table 3:** Expression distribution of antibodies SOX-11, TTF-1, CD56, Syn, and CgA in SCLC.

Number of positive antibodies	Number of cases	Distribution	Positive rate
1	1	Syn+	1.67%
2	2	TTF-1, CD56+	8.33%
	1	CD56, Syn+	
	1	CD56, SOX11+	
	1	Syn, SOX11+	
3	8	TTF-1, CD56, Syn+	21.67%
	1	TTF-1, CD56, CgA+	
	2	TTF-1, CD56, SOX11+	
	1	CD56, Syn, CgA+	
	1	TTF-1, Syn, CgA+	
4	10	TTF-1, CD56, Syn, CgA+	38.33%
	10	TTF-1, CD56, Syn, SOX11+	
	2	TTF-1, CD56, CgA, SOX11+	
	1	TTF-1, Syn, CgA,SOX11+	
5	18	TTF-1, CD56, Syn, CgA, SOX11+	30.00%

## Data Availability

The data used to support the findings of this study are available from the corresponding author upon request.
